This article has been retracted.

# Study on the Macroeconomic Model Based on the Genetic Algorithm

**DOI:** 10.1155/2022/9448895

**Published:** 2022-03-30

**Authors:** Sun Shihao, Yixin Zhou, Yong Wang, Wu Wang

**Affiliations:** ^1^College of Liberal Arts and Social Sciences, City University of Hong Kong, Hong Kong 999077, Hong Kong; ^2^School of Business Economics, Shanghai Business School, Shanghai 201400, China; ^3^Department of Economics, Sejong University, Seoul 05006, Republic of Korea; ^4^Logistics Management, Wuhan Business School, 430056 Wuhan, China

## Abstract

In order to design a more reliable general push time cycle prediction software for macroeconomic indicators, a set of general software is used to serve financial transactions, bulk material transactions, international trade, macro-control and other fields, so as to improve the prediction of macroeconomic indicators. Because the macro data is one-dimensional array data, the essence of the mutation algorithm is to obtain the movement direction of the mutation of data nodes, obtain the distance between the linear programming result and the original data through the least square method, and calculate the average value in the original data, After binary **t**-correction, it refers to the binary **t**-correction results of the one-dimensional matrix before the final evaluation output factor and the one-dimensional matrix after the final evaluation output factor. In this study, genetic algorithm is introduced as the core algorithm. In the algorithm efficiency verification test, the calculation model based on genetic algorithm is constructed in Matlab environment, and the data space construction mode and genetic variation mode of genetic algorithm are explored. Finally, a high-throughput macroeconomic timing prediction scheme based on genetic algorithm is designed. This scheme is more accurate than the paid full-function 10jqka software, and has a higher prediction cycle for stock price and stock index. The simulation software composed of this algorithm has the prediction function that 10jqka software cannot complete.

## 1. Introduction

Economy is a complex system. Micro individuals can interact to determine the form of macro economy, and the dynamics of macro economy will affect the behavior of micro individuals [1]. Foreign research shows that genetic algorithm is an effective tool for complex systems. This method has stable measurement results of macroeconomic uncertainty, consistent with the actual economic operation, can effectively identify economic fluctuations and exogenous shocks, and can accurately reflect the impact degree difference of different shocks [2].

Macroeconomic aggregate, generally using regional gross national product (GDP) or stock market index and other controllable factors to describe macroeconomic state [3]. Commonly used macroeconomic state description data is: regional GDP, regional GDP per capita, monetary nominal purchasing power, iconic main grain price, precious metals and legal currency exchange price, commodity volume and transaction price, stock market index, freight index, etc., conventional macroeconomic state analysis, may be applied to dozens of commonly used macroeconomic state description data [4]. These data mostly expand statistics along the time line, in economics, using time-sharing data and K-line data for statistics. The K-line statistical method is the initial value, final value, highest value, and lowest value in the record statistical period. When the final value is higher than the initial value, it is recorded as the forward K-line, and the reverse K-line when the final value is lower than the initial value.

In this study, a series of macroeconomic models based on genetic algorithm are developed to analyze the stock market trading system, including: the linear programming results are obtained by the least square method. In the analysis, the linear estimation can be obtained for the linear data x, the macro data is a group of dimensional data, and the essence of the mutation algorithm is to obtain the movement direction of the mutation of the data nodes, And the distance between the algorithm obtained by the linear formula and the original data, calculate the average value in the original data, and then undergo binary t-correction, which refers to the binary t-correction results of the one-dimensional matrix before and after adding the final evaluation output factor. In this study, genetic algorithm is introduced as the core algorithm. In the algorithm efficiency verification test, the calculation model based on genetic algorithm is constructed in Matlab environment, and the data space construction mode and genetic variation mode of genetic algorithm are explored. Finally, a high-throughput macroeconomic timing prediction scheme based on genetic algorithm is designed.

In the macroeconomic analysis, it is an important analysis goal to use the previous K-line data to make an early warning or forecast of the K-line data in a certain period of the future [5]. Genetic algorithm was introduced in this study to use certain periodic data as initialization data to obtain more accurate macroeconomic prediction data by obtaining target data for maximum fitness. Using the macroeconomic indicators (GDP) and demographic data, based on the macro vulnerability model and the genetic algorithm, we can also effectively predict and evaluate the economic losses in other emergencies [6].

## 2. Design of the Macroeconomic Genetic Algorithms

The essence of genetic algorithm is to form the determinable original data into data space, take the target data as the target data, use the mutation algorithm to mutate the target data, and finally form the data with the highest evaluation result as the output data. Because the dynamics of complex adaptive systems are usually nonlinear, sometimes even chaotic, it is difficult to obtain accurate analysis results by using traditional linear and fixed-point methods. The algorithm is mainly used for data prediction and analysis with large chaotic effect or unclear data transmission logic. The general mode of genetic algorithm is shown in Figure 1.

For the macroeconomic analysis process, there is a large volume of Basic Data data (most of the original data cycles provided by the platform software are several years to decades), and the analysis and prediction cycle is short (generally need to push the data from 1 to 3 days before). Therefore, the influence of the different raw data selection cycles and the different relevant raw data volume on the accuracy of the final analysis results was explored. The available data structure of the macroeconomic economy is shown in Figure 2.

Combined with the calculation link in Figure 2 above, the following algorithms need to be elaborated.

### 2.1. Linear Planning Algorithm

Linear planning results were obtained by least squares, and in the analysis, for the linear data *X*, linear estimates can be obtained:

(1) $$\begin{array}{c} \hat{\beta }={\left(X^{T}X\right)}^{-1}X^{T}y, \end{array}$$

where *X* is the statistical array data; *X*^*T*^ is the statistics of the last data in the 1D array; and $\hat{\beta }$ is the output data.

### 2.2. Variability Algorithm Based on Target Weights

The essence of the variation algorithm is to obtain the movement direction of data node variation, because the macroeconomic data are 1-dimensional array data, so the movement direction of freedom is only one dimension, obtaining the direction and forward or reverse movement, the algorithm in the previous formula (1), and the distance between the original data calculation average in the original data:

(2) $$\begin{array}{c} ∆x=\frac{\text{Avg}\left(X\right)-\hat{\beta }}{\max\left(X\right)-\min\left(X\right)}, \end{array}$$

where $\hat{\beta }$ is the linear planning results; max(*X*) is the maximum value of the raw data X; min(*X*) is the minimum value of the raw data *X*; Avg(*X*) is the arithmetic average value of the raw data calculated in formula (5); and ∆*x* is the final variation factor of the data variation.

### 2.3. Decision Coefficient *R*^2^ Value Algorithm

In the study design, the determination factor *R*^2^ value and bivariate check *t* value are used to form the evaluation factor, and the final *R*^2^ value and *t* value are considered to reach the output standard, where the *R*^2^ value algorithm is

(3) $$\begin{array}{c} R^{2}=\frac{\beta^{T}X^{T}y-\left(1/n\right)y^{T}uu^{T}y}{\sum_{i=1}^{n}x_{i}^{2}-1/n{\left(\sum_{i=1}^{n}x_{i}\right)}^{2}} \end{array}$$

where *R*^2^ is the decision coefficient evaluation result; other mathematical symbols are found in formula (1) and formula (2).

### 2.4. Bivariate *t* Calibration Algorithm

The *t* test, also known as the bivariate *t* test, is a *t* distribution theory used to infer the probability of differences occurring and thus compare whether the difference between the two mean values is significant. It is mainly suitable for a normal distribution with a small sample size, and the overall standard deviation is unknown. The difference of the data is compared by statistical bivariate *t* calibration method, where the Value value is *t* value. When *t* < 10.000, the smaller statistical difference. Log value is *P* value, statistical reliability is considered when *P* < 0.05, and statistical significance is considered when *P* < 0.01.

The bivariate *t* test designed in this study refers to the results of the bivariate *t* test for adding the one-dimensional matrix before the final evaluation output factor and the one-dimensional matrix after the final evaluation output factor, as shown in

(4) $$\begin{array}{c} t=\frac{\bar{X_{1}}-\bar{X_{2}}}{\sqrt{\left(\left(n_{1}-1\right)\sigma_{1}^{2}+\left(n_{2}-1\right)\sigma_{2}^{2}/n_{1}+n_{2}-2\right)\left(\left(1/n_{1}\right)+\left(1/n_{2}\right)\right)}} \end{array}$$

where $\bar{X_{1}}$, $\bar{X_{2}}$ is the average calculated value of column *X* before and after the final evaluation of the output factor; *σ*_1_^2^, *σ*_2_^2^ is the squared value of the standard deviation of column *X* before and after the final evaluation of the output factor; and *n*_1_, *n*_2_ is the number of column *X* elements before and after adding the final evaluation output factor.

The mean value algorithm is the formula (5):

(5) $$\begin{array}{c} \bar{X}=\overset{n}{\underset{i=1}{\sum }}x_{i}, \end{array}$$

where the meaning of mathematical symbols is the same as the previous formulas;

The standard deviation rate is calculated as

(6) $$\begin{array}{c} \sigma =\frac{1}{n-1}\sqrt{\overset{n}{\underset{i=1}{\sum }}{\left(x_{i}-\bar{X}\right)}^{2}}, \end{array}$$

where the meaning of mathematical symbols is the same as the previous formulas.

## 3. Validation of the Algorithm Efficiency and the Final Algorithm Optimization

In the algorithm efficiency verification test, the genetic algorithm-based computational model is constructed under Matlab, and the final validation results are obtained using the algorithm accuracy. The algorithm accuracy calculates the absolute value between the difference and the actual data, and then calculates the arithmetic average of the ratio, as shown in Equation (7):

(7) $$\begin{array}{c} B=\frac{1}{n}\overset{n}{\underset{i=1}{\sum }}\frac{\left|\hat{x_{i}}-x_{i}\right|}{x_{i}}, \end{array}$$

where *B* is the results of algorithm accuracy evaluation; other mathematical symbols share the previous formulas.

### 3.1. Effect of the Raw Data Cycle on the Prediction Accuracy

In this comparison model, the prediction results of the data of this column supported by a single column data are discussed. Comparing the data of 1 day, 3 days, 7 days and 15 days supported by 1 month to 12 months, respectively, the prediction data travel K-line and form 4 prediction data per day. The final evaluation results are shown in Table 1.

To observe Table 1 data more visually, Table 1 data were visualized to obtain the results of Figure 3:

Observe Table 1 and Figure 3 data. The following data rules were found. The forecast target was 1 or 3 days. High data prediction accuracy can be obtained even with only 1 month of data support. According to the engineering industry consensus on AI data analysis, when the prediction accuracy exceeds 95%, the prediction software has an engineering value. So, under the push-forward prediction period of 1 day ago, select the correlation columns for 2 month data as the base data. Under the push-forward prediction period of 3 days ago, select 3 month data as base data. But under the 7 days and 15 days, it has been impossible to simply increase the amount of relevant data using the algorithm to complete accurate data prediction above 95% accuracy.

### 3.2. The Effect of the Number of Reference Data Columns on the Prediction Accuracy

To further provide the system accuracy under the longer push forward push prediction period requirements, the study assumes hidden conduction logic relationships between other relevant economic data and before the predicted data. For example, there is a hidden transmission logic relationship between bulk material delivery and regional GDP. These relationships are difficult in economics to construct conduction coefficients under statistical models, but the broad association between economic indicators supports genetic algorithms when making forward predictions of certain economic indicator data. Additional data are introduced as the reference data. The raw data space was constructed using the corresponding data columns of the predicted data together with the other data columns, to explore the impact of this approach on the machine learning results of genetic algorithms. The results are shown in Table 2:

To observe Table 2 data more visually, Table 2 data were visualized to obtain the results of Figure 4:

In Figure 4, whether the prediction data of 7 days ago or the forecast data, increase the reference of original data columns, can make the prediction data accuracy is greatly improved, when the reference data column reaches 4 columns, 7 days of prediction accuracy of more than 95%, when the reference data column reaches 6 columns, 5 days of data support prediction accuracy of more than 95%.However, the data in Figure 3 above show that under certain conditions, the accuracy of the macro data prediction and analysis results can exceed 99.9%. For the macroeconomic data prediction results of radical investment projects, the higher the prediction accuracy represents the stronger the risk control ability. Therefore, the study continues to assume that when the reference data column and the original data cycle increase simultaneously, the prediction data accuracy will be more significantly improved. Therefore, in the 15 days before the prediction, different reference data columns and reference data cycles, and the experimental results are obtained in Table 3:

To observe Table 3 data, Table 3 data were visualized to obtain the results of Figure 5:

Observe the data in Table 3 and Figure 5, it is found that increasing the number of reference data columns and the original data cycle can improve the accuracy of pushing data prediction 15 days ago. Taking the 99.9% accuracy threshold as an example, when the original data cycle reaches 7 months and the number of reference data columns reaches 9 columns, 99.9%, while the data cycle reaches 11 months, only 8 columns can reach 99.9%. Data prediction accuracy. It can be seen that increasing the number of reference data columns and the original data cycle can realize the accurate prediction of macroeconomic data.

## 4. The Final Evaluation Ability Test of Macroeconomics by Genetic Algorithms

The application of macroeconomic data prediction software basically focused on the trading platform (stocks, futures, precious metals, etc.) transaction price and comprehensive index prediction, the study uses the genetic algorithm to build the Matlab simulation environment, the original data cycle set to 12 months, related data columns set to 9 columns, push cycle evaluation 1 days, 7 days and 15 days, comparison software for paid version full function flush stock price prediction software (10jqka), from 2000, the algorithm simulation software and reference software, get Table 4

In Table 4, all data have *t* < 10.000, *t* < 0.000 and *P* < 0.01 with significant statistical differences. From the data ratio, the prediction accuracy of the 1-day push prediction period varied, but as the prediction period increased, the two sets of software gradually increased and decreased both *t*-value and *P*-value. We prove that the software has significant algorithm lead in the 10qka period compared with the 10jqka software. The principle of the process is analyzed, because the 10qka prediction method is to construct multiple predictors based on all previous data, and after weighting each index, we form the prediction results. The software focuses more on using machine learning to search for data rules to achieve accurate prediction of data. Moreover, the algorithm can not only realize the prediction of stock price and stock index, but also realize that of other macroeconomic data, as long as the original data can be generated for a long enough time.

## 5. Summary

The development of computer technology makes it possible for us to intelligently simulate the behavior of a monomer in the whole environment. In recent years, the introduction of genetic algorithm in artificial intelligence has applied genetic algorithm to the research of economics. As the core model of macroeconomic forward time cycle prediction, it can achieve high data prediction accuracy and provide data support for macro-control, bulk trading and financial investment with the support of sufficient computing capacity and equipment, However, the algorithm requires high computing power [7]. When most institutions use the algorithm at the same time, the technology leading position of the algorithm will decline. Therefore, using this algorithm can improve the short-term risk control ability of financial institutions, but in the process of economic game, new algorithms still need to be developed.

## Figures and Tables

**Figure 1:** Schematic representation of the general patterns of the genetic algorithm. Basic Data: Basic data provided by the trading platform or the index platform software; Spatial data initialization: Basic data matrix for the Basic Data trip; Target data initialization: Based on the linear planning target data of the Basic Data itinerary, as the data to be varied; Variation: Data variation algorithms, such as the target weight variant algorithm designed in this study; Evaluate: Data evaluation algorithms, such as the weighted evaluation results given by the decision coefficient *R*^2^ used in this study and *t* in the bivariate difference analysis; Loop: Algorithmic cycle branch, re-variant trigger results when poor user data evaluation results; Output & Result: Data analysis results.

**Figure 2:** The raw data acquisition mode and analysis results used in this study. Opening & Maximum & Minimum & Closing: initial value, maximum value, minimum value, final value in K-line data; result of *t*-bivariate *t*-verification, and evaluation value of determination coefficient in *R*^2^ regression analysis.

**Figure 3:** Relationship between raw data volume and prediction accuracy /m=month.

**Figure 4:** Relationship between the number of relevant data columns and the prediction accuracy.

**Figure 5:** Data prediction accuracy was pushed 15 days ago under comprehensive conditions.

**Table 1:** Relationship between raw data volume and prediction accuracy.

Length of basic data	Data prediction cycle			
	1d	3d	7d	15d
1 m	93.69	90.26	63.58	33.29
2 m	98.24	93.71	68.24	38.62
3 m	99.65	95.29	70.13	42.25
4 m	99.87	96.93	71.56	45.78
5 m	99.96	97.82	72.43	47.64
6 m	99.99	98.65	73.11	49.11
7 m	99.99	99.37	73.72	51.59
8 m	99.99	99.54	74.75	52.19
9 m	99.99	99.75	75.63	52.64
10 m	99.98	99.82	76.41	53.16
11 m	99.99	99.91	78.05	53.32
12 m	99.99	99.95	78.44	53.48

d = day; m = month.

**Table 2:** Relationship between the number of relevant data columns and the prediction accuracy.

Number of original data columns	Data prediction cycle	
	3 m-7d	3 m-15d
1	70.13	42.25
2	88.61	63.18
3	93.58	85.27
4	97.42	92.36
5	98.85	94.18
6	99.34	95.35
7	99.63	96.47
8	99.74	97.29
9	99.86	97.94

d = day; m = month.

**Table 3:** The prediction accuracy of 15 days before the push data under the comprehensive conditions.

Number of original data columns	Data prediction cycle(15d)					
	1 m	3 m	5 m	7 m	9 m	11 m
1	33.29	42.25	47.64	51.59	52.64	53.32
2	54.83	63.18	67.24	74.19	82.43	84.29
3	68.76	85.27	87.85	88.65	91.29	92.35
4	86.42	92.36	93.12	94.58	94.36	95.57
5	93.24	94.18	95.28	96.73	97.27	97.69
6	94.15	95.35	97.43	97.92	98.61	98.94
7	95.33	96.47	98.82	99.05	99.36	99.73
8	96.25	97.29	99.53	99.57	99.89	99.99
9	96.18	97.94	99.79	99.98	99.99	99.99

d = day; m = month.

**Table 4:** The forecast accuracy comparison table of stock price and stock index.

Comparison items	1d		7d		15d	
	Price	Index	Price	Index	Price	Index
10jqka	96.27	97.53	85.36	84.17	65.23	63.59
This program	99.99	99.99	99.36	98.97	97.24	96.45
*t*	5.296	4.365	2.138	2.004	0.000	0.000
*P*	0.006	0.005	0.003	0.004	0.001	0.000

## Data Availability

The data underlying the results presented in the study are available within the manuscript.
